# Screening of Medications for Idiopathic Membranous Nephropathy Using Glomerular Whole-Genome Sequencing

**DOI:** 10.1155/2022/9337088

**Published:** 2022-04-14

**Authors:** Yawei Hou, Yameng Li, Wenpu Li, Zhenwei Xiao

**Affiliations:** Shandong University of Traditional Chinese Medicine, Jinan, China

## Abstract

**Objective:**

To explore medications that have a therapeutic effect on idiopathic membranous nephropathy (IMN) using the Gene Expression Omnibus (GEO), the Connectivity Map (CMap) database, and bioinformatics approaches.

**Methods:**

IMN patients' glomerular whole-genome sequencing data were retrieved and screened in the GEO database, differentially expressed genes were identified using GEO2R analysis, a PPI network was built in the STRING database, node degree values were calculated, and topological analysis was performed using the degree value to identify core genes. The WebGestalt database was used to perform GO enrichment and KEGG pathway analyses on the core genes. Candidate medications for the therapy of IMN were collected from the CMap database, and the candidate medications were then searched and analyzed.

**Results:**

113 core genes were identified by topological analysis from the 1157 genes that were shown to be differentially expressed. The enrichment analysis identified several important gene functions and signaling pathways related to IMN. Some possible medications for the treatment of IMN have been found using the CMap database. Naringin, with the lowest CMap score, meaningful *P* value, and specificity score, was predicted as the most likely medication.

**Conclusion:**

The GEO and CMap databases can be used to understand the molecular changes of IMN and to provide new ideas for medication research. However, medication candidates must undergo clinical and experimental testing.

## 1. Introduction

Membranous nephropathy (MN) is a common pathological type of nephrotic syndrome with clinical manifestations of massive proteinuria, hypoalbuminemia, edema, and hyperlipidemia. 70%–80% of MN with an unknown origin is classified as idiopathic membranous nephropathy (IMN). One-third of patients with IMN will eventually develop end-stage renal disease (ESRD), 30% to 40% will resolve spontaneously, and the remainder will have persistent proteinuria with relatively stable renal function [1]. However, these patients are also at an increased risk of life-threatening thromboembolic and cardiovascular events [2]. For extended periods of time, IMN was the second or third largest cause of primary glomerulonephritis resulting in renal failure in the United States and Europe [3]. As a result, IMN imposes a significant financial burden on patients and the healthcare system.

MN may affect people of various nationalities and ethnicities globally. The annual incidence rates of MN in North America are estimated to be 10–12 per million and 2–17 per million in Europe [4–8]. Hormones and immunosuppressants are used to treat [9]. While clinical success can be obtained, there are several complications, including adverse effects, a high likelihood of recurrence upon medication discontinuation, and poor patient compliance. Regardless of the hormone or immunosuppressant used, approximately one-third of people with IMN report no apparent therapeutic benefit [1, 10]. As a result, there is an urgent need to find a medicine that is both effective and safe, with few adverse effects.

System biology studies cells, tissues, and organ systems as systems of interacting components. Methods from systems biology can be applied to the identification of novel medications and the creation of procedures for system pharmacology. And system biology insights can be applied to the development of precision and personalized medical strategies [11]. The Gene Expression Omnibus (GEO) database, a National Center for Biotechnology Information (NCBI) data base for gene expression and hybridization array data, contains a wide assortment of experimental data for various diseases [12, 13]. The GEO database may be used to analyze membranous nephropathy gene expression data. The connectivity map (CMap) database is a resource for understanding the mechanisms of drug action and drug localization using RNA chip technology [14, 15]. If there is a strong negative correlation between the gene expression profile of the sickness and the functional profile of the medication, the medication may have a therapeutic effect on the condition. Medication repositioning or rediscovery refers to the process of relocating or rediscovering existing medications. CMap has been successfully applied in medication rediscovery many times [16–19]. Based on the GEO and CMap databases, this study used system biology methods to screen out the key pathogenic genes and potential therapeutic medications for IMN and provides new ideas for the treatment of IMN. The study flow chart is shown in Figure 1.

## 2. Materials and Methods

### 2.1. Data Sources

The GEO database provided the dataset of membranous nephropathy, and the following screening criteria were used: human glomerular tissue was used as the source of the sample tissue, the normal group had more than three cases, and the illness group had more than thirty. Finally, the dataset GSE108109 was chosen, which is based on the platform GPL19983. GSE108109 was released on May 17, 2018 and was contributed by Grayson et al. [20]. This dataset sequenced the glomerular whole genome of 44 patients with IMN, 30 patients with focal segmental glomerulosclerosis, 16 patients with minimal change disease, 15 patients with ANCA-associated small vessel vasculitis, and 6 healthy people.

### 2.2. Analysis of Differentially Expressed Genes

44 IMN patients in the dataset GSE108109 were assigned as the illness group, while 6 healthy people were set as the control group, and then analyzed using the online analytic tool GEO2R (https://www.ncbi.nlm.nih.gov/geo/geo2r/). We download and filter the findings of the analysis. The screening criteria were adj.*P*.Value < 0.01, ∣Log_2_ Fold Change(FC) | ≥1. And eventually, the differentially expressed genes (DEGs) were determined between IMN and healthy people. The IMN and healthy gene expression matrices were uploaded to the drawing tool Weishengxin (http://www.bioinformatics.com.cn/), and the differentially expressed genes were shown using volcano plots.

### 2.3. Construction and Analysis of the Protein–Protein Interaction Network

The DEGs were uploaded to the STRING database [21], and a network of protein–protein interaction (PPI) with a comprehensive score greater than 0.4 was created. The network that keeps linked nodes was visually analyzed using Cytoscape (version 3.7.2). We calculated the degree value of each node through the Network Analyzer function in the software, and the importance of the node in the network increased with increasing degree value. Referring to previous studies [22, 23], two topological analyses were performed according to the average value of degree. The degree value of each selected node was greater than the overall average value, and the core gene was ultimately obtained.

According to the log_2_FC absolute value of core genes, the top 60 were selected for visual description. To explore the specific regulatory relationships in the PPI network, cluster analysis was performed through the MCODE function of Cytoscape software to calculate node information. The functional modules of the cluster were established according to *K*-Core, and the data parameters were set to the applicable threshold: *K*‐Core > 4.

### 2.4. GO and KEGG Pathway Enrichment Analyses

To clarify the pathogenesis of IMN, the core genes obtained after topological analysis were uploaded to the WebGestalt database. GO and KEGG enrichment analyses were performed on core genes using the WebGestalt database [24, 25]. The results were divided into biological processes (BP), cellular components (CC), molecular functions (MF), and KEGG pathways, which are displayed using bubble charts.

### 2.5. CMap Analysis

The core genes were submitted to the CMap database for research in order to find potential medications for IMN. The CMap database was compiled using the Affymetrix U133A chip [14, 15], and the GSE108109 dataset was compiled using the Affymetrix Human Gene 2.1ST Array. Thus, we needed to convert it through Affymetrix Batch Query (https://www.affymetrix.com/analysis/netaffx/batch_query.affx?netaffx=netaffx4_annot). We saved the converted upregulated and downregulated genes in “.grp” format and uploaded them to the CMap database, respectively. The results, both detailed and permuted, were downloaded. The results were screened according to the mean CMap score, *P* value and specificity of related small molecule compounds, and small molecule compounds that were highly negatively correlated with IMN that may have the potential to treat IMN were screened out.

## 3. Results

### 3.1. Screening of DEGs

We screened 1157 DEGs and discovered that 532 were upregulated, and 625 were downregulated (Figure 2).

### 3.2. Protein–Protein Interactions

The STRING database was used to build the PPI network for DEGs. The PPI network was visualized using Cytoscape. There were 873 nodes and 3982 edges in the network. The core genes were identified after topological analysis (Figure 3). Finally, a disease target network with 113 nodes and 975 edges was constructed, which included 73 upregulated genes and 40 downregulated genes (Figure 4). The core genes were visualized in Figure 5.

By MCODE analysis, 4 modules were extracted from the disease target network, *K*‐Core > 4 (Figure 6). One cluster included 26 nodes and 93 edges (rank 1; score 7.36), one cluster included 35 nodes and 123 edges (rank 2; score 7.235), one cluster included 6 nodes and 14 edges (rank 3; score 5.6), and one cluster included 14 nodes and 30 edges (rank 4; score 4.615).

The colors of the nodes are shown in descending order of Log_2_(FC) from red to blue (with white in the middle). The size of the nodes is described in ascending order of degree value.

### 3.3. GO and KEGG Analyses

To ascertain the link between core genes and IMN, we used the WebGestalt database to conduct GO and KEGG analyses on core genes. BP is mainly associated with the response to endogenous stimuli and the enzyme-linked receptor protein signaling pathway. CC is mainly associated with cell surface and receptor complexes. MF is mainly associated with binding to signaling receptors and protein-containing complexes. The KEGG signaling pathway includes proteoglycan in cancer, PI3K-Akt, MAPK, and other signaling pathways (Figure 7).

### 3.4. CMap Prediction of Potential Medications

We uploaded the core genes to the CMap database, screened small molecule compounds with *P* values and specificity scores, sorted them according to the mean CMap score, and selected the top 10 small molecule compounds. These compounds may be able to reverse the observed IMN gene expression patterns and may be the most promising potential therapeutic agents (Table 1).

## 4. Discussion

Membranous nephropathy is a common pathological type of nephrotic syndrome, and its prevalence is growing in China. A study covering 282 cities and 938 hospitals in China showed that among 71,151 kidney biopsy patients from 2004 to 2014, MN accounted for 23.4%, becoming the second most common pathological type of glomerular disease. Furthermore, the prevalence of MN has grown by 13% every year, whereas the proportion of other major glomerular diseases has remained constant [26]. The 2021 KDIGO practice guidelines recommend 2 treatment regimens: alternating rituximab or cyclophosphamide with corticosteroids and calcineurin inhibitor-based therapy [9]. In clinical practice, it was found that the two treatment options had more side effects and were associated with higher recurrence rates after medications withdrawal. Therefore, there is an urgent need for effective and safe medications for the treatment of IMN. In addition, the economic burden of medications on patients and society should also be considered. As a result, we used bioinformatics analysis methods to screen the key pathogenic genes of IMN and combined them with information from the CMap database to discover potential medications for the treatment of IMN.

MN is a glomerular disease. We screened 1157 DEGs through IMN glomerular whole-genome sequencing data and obtained 113 core genes after topological analysis. The WebGestalt database carried out the KEGG signaling pathway enrichment analysis of core genes, and core genes were mainly related to signaling pathways such as proteoglycan in cancer, PI3K-Akt, and MAPK. The PI3K-Akt and MAPK signaling pathways are closely related to MN. Regulation of autophagy through the PI3K/AKT/mTOR pathway can alleviate MN progression in rat passive Heyman nephritis [27]. Inhibition of the PI3K/AKT/mTOR pathway in human podocytes helps protect podocytes from apoptosis and exerts renal protection. sPLA2-IB can promote podocyte injury by downregulating autophagy by activating the p38 MAPK/mTOR/ULK1 (Ser757) pathway [28]. Single-cell sequencing analysis of renal tissue from healthy individuals and PLA2R-positive IMN patients revealed that differentially expressed genes in renal parenchymal cells lead to MN through pathways such as MAPK [29].

Naringin is a disaccharide derivative that acts as an antitumor agent and an anti-inflammatory agent. The mean CMap score of naringin ranked first and was statistically significant, and naringin was associated with a variety of kidney diseases. In rat renal interstitial fibrosis, naringin attenuates renal interstitial fibrosis [30]. Renal interstitial fibrosis plays an important role in end-stage renal disease (ESRD), and approximately 1/3 of IMN patients will eventually progress to ESRD; thus, naringin may be beneficial to the long-term prognosis of IMN patients. Ischaemia/reperfusion is the main cause of acute renal failure, and naringin can attenuate the expression of Nrf-2 in renal tissue after renal ischemia/reperfusion injury, thereby exerting a renal-protective effect [31]. Naringin attenuates gentamicin-induced renal dysfunction and structural damage in rats through multiple pathways [32]. In streptozotocin- (STZ-) induced diabetic nephropathy rats and high-glucose-induced podocytes, naringin attenuates renal function damage and inhibits podocyte apoptosis in diabetic nephropathy rats by inhibiting NADPH oxidase 4 and in vitro reactive oxygen species levels [33]. Naringin can be used to prevent methotrexate-induced nephrotoxicity by reducing serum creatinine, blood urea nitrogen, and IL-6 [34]. In addition, naringin can reduce nickel-induced nephrotoxicity [35]. In conclusion, naringin has a role in a variety of kidney diseases and has great potential as a medication candidate for the treatment of IMN.

To date, many scholars have verified the reliability of GEO and CMap data mining results through a variety of methods. Zhang et al., through weighted gene coexpression network analysis and the CMap and GEO databases, found that valproic acid and lovastatin may be useful in the treatment of gastric cancer, and the efficacy of the two drugs was verified experimentally [36]. Sirota et al. predicted cimetidine as a candidate drug for the treatment of lung adenocarcinoma and demonstrated its efficacy in vitro and in vivo using mouse models [16].

This research has a few drawbacks. First, the sample size of this study was limited, as there were only 44 IMN patients and 6 healthy people with gene expression data. In addition, no experimental validation or clinical research was conducted on the potential drugs that were the focus of this study. In conclusion, we used the glomerular whole-genome sequencing data of IMN patients, combined with the CMap database, and with the help of bioinformatics analysis methods, we screened the key pathogenic genes of IMN and identified medications with potential therapeutic effects. Animal experiments and clinical trials can be utilized to validate the efficacy of the medications in this investigation.

## Figures and Tables

**Figure 1:** The flow chart for the DEG query signature and the discovery of candidate medications for IMN.

**Figure 2:** DEG volcano map. Volcano plot map showing upregulated and downregulated genes between IMN patients and healthy controls. The horizontal axis represents the value of Log_2_(Fold Change), and the vertical axis represents the value of −Log_10_ (adj.*P*.value). Red represents upregulated genes, blue represents downregulated genes, and gray represents not changed genes.

**Figure 3:** Topological analysis of core genes. (a) IMN-related PPI network made of 873 nodes and 3982 edges. (b) PPI network of important genes extracted from (a). This network is made of 311 nodes and 2388 edges. (c) The core gene PPI network extracted from (b). This network is made of 113 nodes and 975 edges.

**Figure 4:** IMN core gene PPI network. The colors of the nodes are shown in descending order of Log_2_(FC) from red to blue (with white in the middle). The size of the nodes is in ascending order of degree value from small to large.

**Figure 5:** Heatmap of the top 60 core genes by absolute value of Log_2_(FC). The horizontal axis shows the sample name, red represents upregulated genes, and green represents downregulated genes. The colors of the nodes are displayed from red to green (with black in the middle) in descending order of Log_2_(FC).

**Figure 6:** Extraction of modules from disease target networks by MCODE analysis.

**Figure 7:** IMN core genes GO and KEGG pathway enrichment analyses. (a) The BP entry bubble chart of the core gene GO enrichment analysis. (b) The CC entry bubble chart of the core gene GO enrichment analysis. (c) The MF entry bubble of the core gene GO enrichment analysis. (d) The core gene KEGG pathway enrichment analysis bubble plot. Nodes are colored from red to green in descending order of FDR. The size of the nodes is indicated in ascending order of gene counts from small to large. The horizontal axis represents the gene enrichment rate, and the vertical axis represents GO or KEGG entries.

**Table 1:** The 10 most negatively correlated small molecule compounds screened from the CMap database.

Rank	CMap name	Dose	Cell line	Mean CMap score	*P* value	Specificity
9	Naringin	7 *μ*M	PC3	-0.832	0.0298	0.0777
23	Mexiletine	19 *μ*M	PC3	-0.782	0.03681	0.0235
34	Prestwick-1080	15 *μ*M	MCF7	-0.765	0.00147	0
36	PHA-00851261E	10 *μ*M	PC3	-0.761	0.01169	0.0412
50	Pyrantel	11 *μ*M	HL60	-0.739	0.02017	0.0324
52	Pyrimethamine	16 *μ*M	PC3	-0.738	0.01232	0.0467
80	Retrorsine	11 *μ*M	PC3	-0.715	0.03728	0.0769
85	Mecamylamine	20 *μ*M	MCF7	-0.708	0.00096	0
91	Bisoprolol	9 *μ*M	HL60	-0.703	0.02037	0.0055
101	PHA-00851261E	1 *μ*M	MCF7	-0.694	0.01169	0.0412

## Data Availability

All data generated or analyzed during this study are included in this published article. The Chip-seq data have been deposited in the Gene Expression Omnibus database (GEO: GSE108109) (https://www.ncbi.nlm.nih.gov/geo/query/acc.cgi?acc=GSE108109). Requests for material should be made to the corresponding authors.

## References

[1] Dahan K., Debiec H., Plaisier E. (2017). Rituximab for severe membranous nephropathy: a 6-month trial with extended follow-up. *Journal of the American Society of Nephrology: JASN*.

[2] Troyanov S., Wall C. A., Miller J. A., Scholey J. W., Cattran D. C., Toronto Glomerulonephritis Registry Group (2004). Idiopathic membranous nephropathy: definition and relevance of a partial remission. *Kidney International*.

[3] Maisonneuve P., Agodoa L., Gellert R. (2000). Distribution of primary renal diseases leading to end-stage renal failure in the United States, Europe, and Australia/New Zealand: results from an international comparative study. *American Journal of Kidney Diseases: The Official Journal of the National Kidney Foundation*.

[4] Cattran D. C., Brenchley P. E. (2017). Membranous nephropathy: integrating basic science into improved clinical management. *Kidney International*.

[5] De Vriese A. S., Glassock R. J., Nath K. A., Sethi S., Fervenza F. C. (2017). A proposal for a serology-based approach to membranous nephropathy. *Journal of the American Society of Nephrology*.

[6] Kumar V., Ramachandran R., Kumar A. (2015). Antibodies to m-type phospholipase A2 receptor in children with idiopathic membranous nephropathy. *Nephrology*.

[7] Debiec H., Ronco P. (2014). Immunopathogenesis of membranous nephropathy: an update. *Seminars in Immunopathology*.

[8] McGrogan A., Franssen C. F., de Vries C. S. (2011). The incidence of primary glomerulonephritis worldwide: a systematic review of the literature. *Nephrology, Dialysis, Transplantation*.

[9] Rovin B. H., Adler S. G., Barratt J. (2021). Executive summary of the KDIGO 2021 guideline for the management of glomerular diseases. *Kidney International*.

[10] Couser W. G. (2017). Primary membranous nephropathy. *Clinical Journal of the American Society of Nephrology*.

[11] Tavassoly I., Goldfarb J., Iyengar R. (2018). Systems biology primer: the basic methods and approaches. *Essays in Biochemistry*.

[12] Edgar R., Domrachev M., Lash A. E. (2002). Gene Expression Omnibus: NCBI gene expression and hybridization array data repository. *Nucleic Acids Research*.

[13] Barrett T., Wilhite S. E., Ledoux P. (2013). NCBI GEO: archive for functional genomics data sets--update. *Nucleic Acids Research*.

[14] Lamb J., Crawford E. D., Peck D. (2006). The Connectivity Map: using gene-expression signatures to connect small molecules, genes, and disease. *Science (New York, N.Y.)*.

[15] Subramanian A., Narayan R., Corsello S. M. (2017). A next generation connectivity map: L1000 platform and the first 1,000,000 profiles. *Cell*.

[16] Sirota M., Dudley J. T., Kim J. (2011). Discovery and preclinical validation of drug indications using compendia of public gene expression data. *Science Translational Medicine*.

[17] Qu X. A., Rajpal D. K. (2012). Applications of Connectivity Map in drug discovery and development. *Drug Discovery Today*.

[18] Kunkel S. D., Suneja M., Ebert S. M. (2011). mRNA expression signatures of human skeletal muscle atrophy identify a natural compound that increases muscle mass. *Cell Metabolism*.

[19] Hassane D. C., Guzman M. L., Corbett C. (2008). Discovery of agents that eradicate leukemia stem cells using an in silico screen of public gene expression data. *Blood*.

[20] Grayson P. C., Eddy S., Taroni J. N. (2018). Metabolic pathways and immunometabolism in rare kidney diseases. *Annals of the Rheumatic Diseases*.

[21] Szklarczyk D., Gable A. L., Nastou K. C. (2021). The STRING database in 2021: customizable protein-protein networks, and functional characterization of user-uploaded gene/measurement sets. *Nucleic Acids Research*.

[22] Zhang Y., Li Z., Yang M. (2013). Identification of GRB2 and GAB1 coexpression as an unfavorable prognostic factor for hepatocellular carcinoma by a combination of expression profile and network analysis. *PLoS One*.

[23] Wang S., Wang H., Lu Y. (2017). Tianfoshen oral liquid: a CFDA approved clinical traditional Chinese medicine, normalizes major cellular pathways disordered during colorectal carcinogenesis. *Oncotarget*.

[24] Liao Y., Wang J., Jaehnig E. J., Shi Z., Zhang B. (2019). WebGestalt 2019: gene set analysis toolkit with revamped UIs and APIs. *Nucleic Acids Research*.

[25] Wang J., Vasaikar S., Shi Z., Greer M., Zhang B. (2017). WebGestalt 2017: a more comprehensive, powerful, flexible and interactive gene set enrichment analysis toolkit. *Nucleic Acids Research*.

[26] Xu X., Wang G., Chen N. (2016). Long-term exposure to air pollution and increased risk of membranous nephropathy in China. *Journal of the American Society of Nephrology: JASN*.

[27] Di Tu Q., Jin J., Hu X., Ren Y., Zhao L., He Q. (2020). Curcumin improves the renal autophagy in rat experimental membranous nephropathy via regulating the PI3K/AKT/mTOR and Nrf2/HO-1 signaling pathways. *BioMed Research International*.

[28] Yang L., Wu Y., Lin S. (2021). sPLA2-IB and PLA2R mediate insufficient autophagy and contribute to podocyte injury in idiopathic membranous nephropathy by activation of the p38MAPK/mTOR/ULK1ser757 signaling pathway. *FASEB sournal*.

[29] Xu J., Shen C., Lin W. (2021). Single-cell profiling reveals transcriptional signatures and cell-cell crosstalk in anti-PLA2R positive idiopathic membranous nephropathy patients. *Frontiers in Immunology*.

[30] Wang R., Wu G., Dai T. (2021). Naringin attenuates renal interstitial fibrosis by regulating the TGF-*β*/Smad signaling pathway and inflammation. *Experimental and Therapeutic Medicine*.

[31] Amini N., Sarkaki A., Dianat M., Mard S. A., Ahangarpour A., Badavi M. (2019). Protective effects of naringin and trimetazidine on remote effect of acute renal injury on oxidative stress and myocardial injury through Nrf-2 regulation. *Pharmacological Reports*.

[32] Sahu B. D., Tatireddy S., Koneru M. (2014). Naringin ameliorates gentamicin-induced nephrotoxicity and associated mitochondrial dysfunction, apoptosis and inflammation in rats: possible mechanism of nephroprotection. *Toxicology and Applied Pharmacology*.

[33] Zhang J., Yang S., Li H., Chen F., Shi J. (2017). Naringin ameliorates diabetic nephropathy by inhibiting NADPH oxidase 4. *European Journal of Pharmacology*.

[34] Elsawy H., Alzahrani A. M., Alfwuaires M., Abdel-Moneim A. M., Khalil M. (2021). Nephroprotective effect of naringin in methotrexate induced renal toxicity in male rats. *Biomedicine & Pharmacotherapy*.

[35] Amudha K., Pari L. (2011). Beneficial role of naringin, a flavanoid on nickel induced nephrotoxicity in rats. *Chemico-Biological Interactions*.

[36] Zhang L., Kang W., Lu X., Ma S., Dong L., Zou B. (2019). Weighted gene co-expression network analysis and connectivity map identifies lovastatin as a treatment option of gastric cancer by inhibiting HDAC2. *Gene*.

